The article "Random Walk Algorithm-Based Computer Tomography (CT) Image Segmentation Analysis Effect of Spiriva Combined with Symbicort on Immunologic Function of Non-Small-Cell Lung Cancer" was published in 2022. Journal: Comput Math Methods Med.

# Random Walk Algorithm-Based Computer Tomography (CT) Image Segmentation Analysis Effect of Spiriva Combined with Symbicort on Immunologic Function of Non-Small-Cell Lung Cancer

**DOI:** 10.1155/2022/1986647

**Published:** 2022-06-03

**Authors:** Xiaodan Li, Wei Liu, Mianjie Liang, Zengtao Sun

**Affiliations:** ^1^Department of Respiratory, The Second Affiliated Hospital of Tianjin University of Traditional Chinese Medicine, Tianjin 300000, China; ^2^Department of Respiratory, Graduate School of Tianjin University of Traditional Chinese Medicine, Tianjin 301617, China; ^3^Department of Respiratory, Tianjin University of Traditional Chinese Medicine, Tianjin 301617, China

## Abstract

The objective of this research was to explore the effect of the treatment regimen of Spiriva combined with Symbicort on the immune function of non-small-cell lung cancer (NSCLC) based on computed tomography (CT) imaging features. An automatic CT image segmentation algorithm (RW-CT) was constructed based on random walk (RW) and image segmentation technology. The image segmentation algorithm based on the Toboggan method (C-CT) was introduced to compare with the traditional RW algorithm. 60 subjects were divided into four groups: a Chinese combined with Western medicine group (treated with Spiriva combined with Symbicort, group C+W), a Chinese medicine group (treated with Spiriva, group C), a Western medicine group (treated with Symbicort, group W), and a model group for control (group M). The results show that the Dice coefficient of the RW-CT algorithm was obviously larger than that of the C-CT algorithm and the RW algorithm, while the Hausdorff distance (HD) of the RW-CT algorithm was much smaller than that of the other two algorithms (*P* < 0.05). The proportion of positive cells of hypoxia-inducible factor-1*α* (HIF-1*α*) in group C+W was the least (15%-23%), followed by the group W (21%-29%) and the group C (28%-37%), and that in the group M was the highest (39%-49%). There was a remarkable difference in the immunohistochemical scores (HIS) of vascular endothelial growth factor (VEGF) in the tumor tissues between group C+W and the group M (*H* = 14.200, *P* = 0.001), but there was no great difference from the group C and the group W (*P* > 0.05). There was a notable difference in the IHS of vascular endothelial factor recepto-2 (VEGFR-2) between the group C+W medication group and the group M (*H* = 12.800, *P* = 0.002), and there was no statistical difference between the group C and W (*P* > 0.05). In short, the RW-CT constructed based on RW was better than the traditional algorithms for CT image segmentation. The Spiriva combined with Symbicort could effectively inhibit the expression of VEGF, VEGFR-2, and HIF-1*α* in NSCLC and promote the immunologic function of the body.

The article "Random Walk Algorithm-Based Computer Tomography (CT) Image Segmentation Analysis Effect of Spiriva Combined with Symbicort on Immunologic Function of Non-Small-Cell Lung Cancer" was published in 2022. Journal: Comput Math Methods Med.

## 1. Introduction

Lung cancer is one of the most common malignant tumors worldwide and has become the first cause of death from malignant tumors in the urban population in China. In addition, the lung cancer mainly includes the NSCLC and small-cell lung cancer [1, 2]. Among them, the cancer cells of NSCLC are large and irregular in shape under the microscope, and its incidence can account for about 85% of the total number of lung cancers. It is a kind of cancer with relatively mild disease, mainly including three cell subtypes: adenocarcinoma, squamous cell carcinoma, and large cell carcinoma. It is clinically manifested as fatigue, weight loss, decreased appetite, difficulty breathing, coughing, chest pain, hemoptysis, and other symptoms [3]. The specific cause of NSCLC is still unclear, but it is generally believed to be related to smoking, genetic factors, ionizing radiation, air pollution, and radioactive metal dust. Since there are no any obvious symptoms for NSCLC in the early stage, it is easy to be misdiagnosed as pneumonia or pneumothorax, so that the treatment is delayed. When it is diagnosed, it may have developed to the middle and late stage, and the survival rate of the patients is greatly reduced [4, 5]. At present, oral and injection (intravenous or intramuscular) drugs are mainly used clinically to kill cancer cells throughout the body, such as Aquatra, Spiriva, Symbicort, and Seretide [6].

With the development of imaging, NSCLC often is diagnosed with X-rays, CT images, and mediastinoscopy in clinic. Of which, X-rays can understand the location and size of lung cancer, as well as local emphysema and atelectasis caused by bronchial obstruction, but the resolution is low and easy to misdiagnose [7, 8]. Mediastinoscopy is mainly used for patients with mediastinal lymph node metastasis and is not suitable for surgical treatment, while other methods cannot obtain pathological diagnosis [9]. CT imaging can detect the bone metastases earlier, with high resolution, easy operation, and low cost. It occupies an important position in the impact of lung cancer. RW is a mathematical form similar to Brownian motion, used to express the irregular changes. It is like a person walking on the street; there are no rules to know where is his next move [10–12]. This theory is also widely cited and used in medical image processing. An image can be regarded as composed of a certain number of points and edges, and the region can be segmented to extract key information [13]. Graph cut algorithm is a very useful and popular energy optimization algorithm. It is widely used in the field of image processing, such as background segmentation, stereo vision, and matting. At present, it is widely used in the field of medical images. Therefore, the RW theory was intended to be adopted to construct a CT image segmentation algorithm to explore the therapeutic effect of Spiriva combined with Symbicort on NSCLC.

The article "Random Walk Algorithm-Based Computer Tomography (CT) Image Segmentation Analysis Effect of Spiriva Combined with Symbicort on Immunologic Function of Non-Small-Cell Lung Cancer" was published in 2022. Journal: Comput Math Methods Med.

In summary, an automatic CT image segmentation algorithm (RW-CT) was constructed based on RW. The image segmentation algorithm C-CT based on the Toboggan method was introduced to compare with the traditional RW algorithm and applied to 60 cases of NSCLC for analysis of drug treatment effects in mice with lung cancer. The positive expressions of HIF-1*α*, VEGF, and VEGFR-2 in the three groups of mice were compared to explore the effect of Spiriva combined with Symbicort on the immunologic function of mice with NSCLC.

The structure of this study was as follows. Firstly, an image segmentation algorithm based on random walk was constructed and compared with the CT image segmentation algorithm based on Toboggan and the traditional random walk algorithm to analyze the performance in terms of Dice coefficient and Hausdorff distance. Secondly, 60 healthy male BALB/c nude mice were selected as research samples, and a mouse model of non-small-cell lung cancer was constructed, and the mice were divided into four groups: a Chinese combined with Western medicine group (treated with Spiriva combined with Symbicort, group C+W), a Chinese medicine group (treated with Spiriva, group C), a Western medicine group (treated with Symbicort, group W), and a model group for control (group M). Thirdly, immunohistochemical staining was used to detect the levels of HIF-1*α*, VEGF, and VEGFR-2 in mice after treatment; and the image segmentation performances of the three algorithms were discussed, and the results of immunohistochemical staining were discussed. Finally, the research conclusions, shortcomings, and future prospects of this article were analyzed and given.

## 2. Materials and Methods

### 2.1. Research Animals

Sixty healthy male BALB/c nude mice that were bred for 6-8 weeks were selected as the research objects, with a weight range of 20-22 g. They were raised in an environment with a temperature of about 25°C and regularly fed sterile food and water every day. Based on the different dosing regimens, they were divided into group C+W (treated with Spiriva combined with Symbicort), group C (treated with Spiriva), group W (treated with Symbicort), and group M (model control). The experiment was developed in accordance with the experimental protocol and standardized operating procedures strictly, without violating the ethical requirements.

The article "Random Walk Algorithm-Based Computer Tomography (CT) Image Segmentation Analysis Effect of Spiriva Combined with Symbicort on Immunologic Function of Non-Small-Cell Lung Cancer" was published in 2022. Journal: Comput Math Methods Med.

### 2.2. Construction of a Mouse Model of Non-Small-Cell Lung Cancer

Firstly, the mouse Lewis lung cancer cells were cultured in 10% fetal bovine serum culture medium and then cultured in 5% CO_2_ at 37°C. The culture medium was replaced every 3 days. When the number of viable cells grew to 90%, the culture could be stopped and a suspension should be prepared. Then, all the mice were inoculated subcutaneously at the back of the axillary line and each with 0.2 mL lung cancer cells. When the cell count was 5 × 10^6^ cells/mL, the NSCLC mouse model was obtained successfully.

### 2.3. CT Scanning

64 CT scanner was adopted to examine the mice. The mouse was placed in a supine position, and resting tomography was performed from the middle of the mouse femur to the head position, and data of 8 mice were collected. The scanning parameters were defined as follows: the voltage was 120 kV, the current was 140 mA, the pitch was 0.85, and the layer thickness was 5 mm. After the scan was completed, the image was transferred to the workstation for segmentation and reconstruction.

### 2.4. Image Segmentation Algorithm Based on Random Walk

In the RW theory, an image could be composed of a certain number of points and edges. It was assumed that an image could be mapped to a weighted graph, so the below equation could be obtained:

(1) $$\begin{array}{c} T=\left(W,F\right). \end{array}$$

In equation (1), *T* represented the weighted graph, *W* represented the node range, and *F* referred to the boundary range. A node in the image was set to *w*, and an edge was set to *f*, and then *w* ∈ *W* and *f* ∈ *W* × *W*. The weight of the edge belonged to the gray-scale mapping of the image, so the Gaussian weight function was introduced to express, as shown below:

(2) $$\begin{array}{c} v_{ij}=\exp\left(-\beta {\left(t_{i}-t_{j}\right)}^{2}\right). \end{array}$$

In equation (2), *t*_*i*_ represented the brightness of the pixel *w*_*i*_, *β* referred to the weight coefficient, and *v*_*ij*_ indicated the probability of a random walk through the edge *f*_*ij*_. Considering that the probability solution problem was similar to the Dirichlet integral problem, so it was transformed into

(3) $$\begin{array}{c} G\left(o\right)=\frac{1}{2}\int {\left|\nabla o\right|}^{2}d\Omega . \end{array}$$

In equation (3), *G*(*o*) was the integral of *o*, ∇*o* referred to the harmonic function, and *Ω* indicated the image area. The harmonic function could satisfy the Laplace's equation, and then, the Dirichlet integral problem can be converted into a harmonic function for solving boundary conditions. The equation was as follows:

(4) $$\begin{array}{c} \nabla^{2}o=0. \end{array}$$

Thus, the Laplace matrix could be expressed as below:

(5) $$\begin{array}{c} P_{ij}=\left\{\begin{array}{cc} d_{i}, & i={jw}_{i},\\ -v_{ij}, & w_{i}\text{ adjacent }w_{j},\\ 0, & \text{others}. \end{array}\right. \end{array}$$

In equation (5), *P*_*ij*_ referred to the vertex guided by *w*_*i*_ and *w*_*j*_, and *d*_*i*_ represented the degree of a specific node. Then, the incidence matrix of the specific edge and point can be supposed as

(6) $$\begin{array}{c} B_{f_{ij}w_{k}}=\left\{\begin{array}{cc} +1, & \text{if }i=k,\\ -1, & \text{if }j=k,\\ 0, & \text{others}, \end{array}\right. \end{array}$$

where *B*_*f*_*ij*_*w*_*k*__ was determined by *f*_*ij*_ and *f*_*i*_ jointly. Therefore, it was necessary to find a cut with the least cost to complete the image segmentation process for a weighted image. The image segmentation algorithm was introduced in this study for processing, and the two special points of the image were, respectively, *Q* and *I*, respectively. Thus, below equation could be obtained:

(7) $$\begin{array}{c} W=P\cup \left[Q,I\right]. \end{array}$$

In equation (7), *P* represented a collection of pixels. The edges in the image can be divided into edges connecting the vertices and endpoints of the image and edges connecting the pixels to the terminal nodes. Then, the set of edges could be expressed as below:

(8) $$\begin{array}{c} F=N\cup \left\{\left[\theta ,S\right],\left[\theta ,I\right]\right\}. \end{array}$$

In equation (8), *N* represented the connected neighborhood, *θ* referred to the pixel point, and *S* stood for the terminal node. Therefore, the final result of image segmentation can be obtained as long as the set of all cut edges of the image was found and the sum of the weights of the edges was minimized.

The article "Random Walk Algorithm-Based Computer Tomography (CT) Image Segmentation Analysis Effect of Spiriva Combined with Symbicort on Immunologic Function of Non-Small-Cell Lung Cancer" was published in 2022. Journal: Comput Math Methods Med.

### 2.5. Algorithm Performance Evaluation Index

The image segmentation algorithm RW-CT optimized with RW was compared with the CT image segmentation algorithm C-CT based on the Toboggan method and the traditional RW. The Dice coefficient and Hausdorff distance (HD) were adopted as indicators to evaluate the algorithm performances.

1. The Dice coefficient could judge the quality of the segmentation result according to the degree of overlap between the segmentation result and the gold standard. The size was [0,1], and the larger the value, the better the segmentation effect, as given below:

(9) $$\begin{array}{c} \text{Dice}=2\frac{\left|R_{1}\cap R_{2}\right|}{\left|R_{1}\right|+\left|R_{2}\right|}. \end{array}$$

In equation (9), *R*_1_ represented the segmentation result, and *R*_2_ referred to the gold standard

(2) Hausdorff distance displayed the maximum distance in the minimum set of all voxel point distances in the two segmentation results. The equation was as follows:

(10) $$\begin{array}{c} \text{HD}=\underset{a\in R^{\#}}{\max}\left[d\left(a,R^{*}\right),d\left(a,R^{*}\right)\right]. \end{array}$$

In equation (10), *R*^∗^ and *R*^#^ represent two segmentation results, respectively, and *d*(*a*, *R*^∗^) referred to the distance from *R*^#^ to *R*^∗^

The article "Random Walk Algorithm-Based Computer Tomography (CT) Image Segmentation Analysis Effect of Spiriva Combined with Symbicort on Immunologic Function of Non-Small-Cell Lung Cancer" was published in 2022. Journal: Comput Math Methods Med.

### 2.6. Immunohistochemical Staining

The immunohistochemical staining was used to detect the levels of HIF-1*α*, VEGF, and VEGFR-2 after treatment in mice. The specific steps were defined as follows: the lung tissue was fixed, embedded, sliced, and then dried at 60°C for later use; it was repaired with microwave and washed three times with phosphate buffer solution (PBS); it was incubated with 3% deionized water for 15 minutes, washed three times with PBS, and added with the diluted primary antibody FGF-2 for overnight at 4°C; it was added with polymer adjuvant to incubate for 20 minutes, washed 3 times again with PBS, and then added with biotin-labeled anti-rabbit polymer for 30 minutes at 37°C; it was added with 3,3′-diaminobenzidine to develop color for 30 minutes, rinsed with tap water, and sealed with neutral gum. 10 high-definition field of view areas had to be selected under high-definition Olympus microscope to observe and record the positive cells and calculate the HIS.

### 2.7. Statistical Methods

The data processing was analyzed by SPSS19.0 version statistical software, the measurement data and the count data were expressed as mean ± standard deviation ($\overset{¯}{x}\pm s$) and percentage (%), respectively. The Dice coefficients of RW-CT, C-CT, and RW algorithms were compared by independent *t* test. The IHS of HIF-1*α*, VEGF, and VEGFR-2 was compared by analysis of variance. The difference was statistically meaningful at *P* < 0.05.

## 3. Results

### 3.1. CT Images of Mice Model with Non-Small-Cell Lung Cancer

Figure 1 shows a lung CT image a mouse (weighted 20 g). The pulmonary window showed the patch and strip shadow tuberculosis foci in the right upper lung, fibrous proliferative tuberculosis, and the eccentric hollow in the left upper lung with nodules inside (Figure 1(a)); the mediastinal window showed calcification in the right upper pulmonary tuberculosis foci and the mass with uniform density in the right upper lung (Figure 1(b)).

### 3.2. Evaluation on Segmentation Performances of the Three Algorithm

Figure 2 illustrates the evaluation indicators for segmentation performances of the three algorithms. It could be observed that Dice coefficient and HD of the C-CT algorithm were 7.31 and 10.62, respectively; those of the RW algorithm were 7.02 and 11.35, respectively; and those of RW-CT algorithm were 8.96 and 6.43, respectively. Among them, the Dice coefficient of the RW-CT algorithm was much increased in contrast to that of the C-CT algorithm and the RW algorithm with statistically significance (*P* < 0.05); the HD of the RW-CT algorithm was much smaller than that of the other algorithms with substantial significance (*P* < 0.05).

The article "Random Walk Algorithm-Based Computer Tomography (CT) Image Segmentation Analysis Effect of Spiriva Combined with Symbicort on Immunologic Function of Non-Small-Cell Lung Cancer" was published in 2022. Journal: Comput Math Methods Med.

### 3.3. Immunohistochemical Staining Result for IHS of HIF-1*α* in the Four Groups of Mouse Tumor Tissues

Figure 3 discloses the immunohistochemical staining results of HIF-1*α* of tumor tissues in the four groups of mice. The colors corresponding to group M, W, C, and C+W were black brown, brown, black brown with little brown, and light yellow with little brown, respectively; and the proportion of positive cells in these groups was 39%-49%, 21%-29%, 28%-37%, and 15%-23%, respectively.

As shown in Table 1, independent sample K-W test was adopted for comparing the IHS of HIF-1*α* among the group M, W, C, and C+W, and the results showed that the difference was statistically meaningful (*H* = 15.472, *P* = 0.001).

After Bonferroni correction, the IHS scores of HIF-1*α* between group C+W and group C, between group C+W and group M, and between group W and group M were obviously meaningful (*H* = 9.400, *P* = 0.033; *H* = 11.200, *P* = 0.006; and *H* = 9.000, *P* = 0.047, respectively).

The IHS scores of HIF-1*α* in tumor tissue of mice between the group C+W and W, between the group W and C, and between the group C and M were different without statistical significance (*H* = 2.200, *P* = 1.000; *H* = 7.200, *P* = 0.201; and *H* = 1.800, *P* = 1.000, respectively).

The IHS scores of HIF-1*α* in tumor tissue of mice could be ordered as group M > C > W > C+W (from top high to low).

### 3.4. Immunohistochemical Staining Result for HIS of VEGF in the Four Groups of Mouse Tumor Tissues

As shown in Figure 4, the immunohistochemical staining results of VEGF in mouse tumor tissue showed that the color of group M was black brown, and the proportion of positive cells was 29%-35%; the color corresponding to group W was mainly brown with light yellow, and the proportion of positive cells was 17%-25%; the color corresponding to group C was mainly brown with a small amount of brown, and the proportion of positive cells was 21%-29%; and the color of group C+W was light yellow, and the proportion of positive cells was 7%-15%.

The proportion of HIF-1*α*-positive cells in tumor tissues of mice in the four groups was compared (Figure 5). The proportion of HIF-1*α*-positive cells in tumor tissues of mice in group M was significantly higher than that in group C, group C+W, and group W, and the difference was statistically significant (*P* < 0.05); the proportion of HIF-1*α*-positive cells in tumor tissues of mice in group C+W was significantly lower than that in group C and group W, and the difference was statistically significant (*P* < 0.05).

The article "Random Walk Algorithm-Based Computer Tomography (CT) Image Segmentation Analysis Effect of Spiriva Combined with Symbicort on Immunologic Function of Non-Small-Cell Lung Cancer" was published in 2022. Journal: Comput Math Methods Med.

Table 2 shows the comparison on the IHS of VEGF among the group M, W, C, and C+W after the independent sample K-W test, and the results showed that the difference was statistically meaningful (*H* = 16.505, *P* = 0.001).

After Bonferroni correction, the IHS scores of VEGF between group C+W and group M were obviously meaningful (*H* = 14.200, *P* = 0.001).

The IHS scores of VEGF in tumor tissue of mice between the group C+W and W, between the group C+W and C, between the group W and C, and between the group W and M were different without statistical significance (*H* = 6.000, *P* = 0.548; *H* = 8.600, *P* = 0.093; *H* = 2.600, *P* = 1.000; *H* = 8.200, *P* = 0.126; and *H* = 5.600, *P* = 0.691, respectively).

The IHS scores of VEGF in tumor tissue of mice could be ordered as group M > C > W > C+W (from top high to low).

### 3.5. Immunohistochemical Staining Result for HIS of VEGFR-2 in the Four Groups of Mouse Tumor Tissues

In the immunohistochemical staining, the result for VEGFR-2 in tumor tissue of mice is given in Figure 6. It suggested that the colors in group M and W were black brown and brown with light yellow, respectively, and the positive cells accounted for 29%-35% and 17%-25%, respectively; colors in group C and C+W were brown with black brown and light yellow, respectively, and the positive cells accounted for 21%-29% and %-15%, respectively.

The proportion of VEGF-positive cells in tumor tissues of mice in the four groups was compared (Figure 7). The proportion of VEGF-positive cells in tumor tissues of mice in group M was significantly higher than that in group C, group C+W, and group W, and the difference was statistically significant (*P* < 0.05); the proportion of VEGF-positive cells in tumor tissues of mice in group C+W was significantly lower than that in group C and group W, and the difference was statistically significant (*P* < 0.05).

Table 3 showed the comparison on the IHS of VEGFR-2 among the group M, W, C, and C+W after the independent sample K-W test, and the results showed that the difference was statistically meaningful (*H* = 14.617, *P* = 0.002).

After Bonferroni correction, the IHS scores of VEGFR-2 between group C+W and group M were obviously meaningful (*H* = 12.800, *P* = 0.002). The IHS scores of VEGFR-2 in tumor tissue of mice between the group C+W and W, between the group C+W and C, between the group W and C, between the group W and M, and between the group C+W and M were different without statistical significance.

The article "Random Walk Algorithm-Based Computer Tomography (CT) Image Segmentation Analysis Effect of Spiriva Combined with Symbicort on Immunologic Function of Non-Small-Cell Lung Cancer" was published in 2022. Journal: Comput Math Methods Med.

The IHS scores of VEGFR-2 in tumor tissue of mice could be ordered as group M > C > W > C+W (from top high to low).

## 4. Discussion

NSCLC is currently one of the major malignant tumors that endanger people's lives and health, and its morbidity and mortality have risen dramatically with the improvement of living standards. Unfortunately, there are no clear symptoms in early NSCLC, which makes clinical diagnosis and treatment not timely. Therefore, an image segmentation algorithm RW-CT was proposed based on the RW, and the image segmentation algorithm C-CT based on the Toboggan method was introduced to compare with the traditional RW algorithm. The results showed that the Dice coefficient and HD of the RW-CT algorithm were observably larger and smaller than those of the C-CT algorithm and the RW algorithm, respectively (*P* < 0.05), which was similar to the research result of Song et al. [14]. It indicated that the RW-CT algorithm constructed was better than C-CT algorithm and RW algorithm for CT image segmentation, so its applicability was high. Then, the RW-CT algorithm was applied to the analysis of the drug treatment effect of 60 NSCLC mice. The results revealed that in the HIF-1*α* staining results, the proportion of HIF-1*α*-positive cells in tumor tissues of mice in group M was significantly higher than that in group C, group C+W, and group W; the proportion of HIF-1*α*-positive cells in tumor tissues of mice in group C+W was significantly lower than that in group C and group W, and the difference was statistically significant (*P* < 0.05). HIF-1*α* is closely related to the growth, invasion, and metastasis of tumor tissues, and it is also a transcriptional regulator that plays an important role in tumor hypoxia [15]. The results in this study showed that both Spiriva combined with Symbicort and single Spiriva or Symbicort could reduce the expression of HIF-1*α* in NSCLC mice, and Spiriva combined with Symbicort had the best improvement effect.

In addition, it was also found that the difference in the IHS score in VEGF between group C+W and M mouse tumor tissue was dramatically visible (*H* = 14.200, *P* = 0.001), but there was no statistical difference between group C and W (*P* > 0.05). The proportion of VEGF-positive cells in tumor tissue of mice in group C+W was significantly lower than that in group C and group W, and the difference had statistical significance (*P* < 0.05). As the most important immunosuppressive factor, VEGF exerts an important role in the formation and occurrence of tumors. The above results indicated that Spiriva combined with Symbicort could effectively reduce the VEGF levels and promote the immunologic function of NSCLC and has the best promotion effect [16]. There was a huge difference in the IHS score in VEGFR-2 in tumor tissue between group C+W and M (*H* = 12.800, *P* = 0.002), but there was no statistical difference between group C and W (*P* > 0.05). It was similar to the results of Jiang et al. [17], who found that VEGFR-2 also played a key role in tumor formation, indicating that Spiriva combined with Symbicort could effectively reduce the level of VEGFR-2 and promote the immunologic function of NSCLC.

The article "Random Walk Algorithm-Based Computer Tomography (CT) Image Segmentation Analysis Effect of Spiriva Combined with Symbicort on Immunologic Function of Non-Small-Cell Lung Cancer" was published in 2022. Journal: Comput Math Methods Med.

## 5. Conclusion

An RW-CT was established based on the RW, and C-CT based on the Toboggan method and the traditional RW algorithm were introduced for comparison. They were applied to 60 mice with NSCLC to analyze and compare the drug treatment effect. It was found that the image segmentation algorithm RW-CT constructed based on random walk is superior to the traditional algorithm in the segmentation of CT images. Spiriva combined with Symbicort could effectively reduce the expression levels of VEGF, VEGFR-2, and HIF-1*α* in mice with NSCLC, thereby promoting the immune cell function. However, the sample size of mice selected was small, which may have a certain impact on the results. In the follow-up, it will consider increasing the animal sample size and further explore the effect of Spiriva combined with Symbicort on NSCLC. In conclusion, the use of artificial intelligence algorithms and imaging techniques provides a scientific reference for the clinical diagnosis and treatment of lung cancer.

## Figures and Tables

**Figure 1:** A lung CT image of a mouse (weighted 20 g). (a) showed the CT from pulmonary window. (b) showed the CT from mediastinal window.

**Figure 2:** Evaluation indicators for segmentation performance of the three algorithms. (a) and (b) illustrated the Dice coefficient and HD of the algorithms, respectively. ^∗^Compared with RW-CT algorithm, *P* < 0.05.

**Figure 3:** Immunohistochemical staining result for IHS of HIF-1*α* in the four groups of mouse tumor tissues (×400). (a)–(d) showed the results of group C, C+W, M, and W, respectively.

**Figure 4:** Immunohistochemical staining result for IHS of VEGF in the four groups of mouse tumor tissues (×400). (a)–(d) showed the results of group C, C+W, M, and W, respectively.

**Figure 5:** Proportion of HIF-1*α*-positive cells in tumor tissues of mice in the four groups. ^∗^Compared with group M, *P* < 0.05; ^#^compared with group C+W, *P* < 0.05.

**Figure 6:** Immunohistochemical staining result for IHS of VEGFR-2 in the four groups of mouse tumor tissues (×400). (a)–(d) showed the results of group C, C+W, M, and W, respectively.

The article "Random Walk Algorithm-Based Computer Tomography (CT) Image Segmentation Analysis Effect of Spiriva Combined with Symbicort on Immunologic Function of Non-Small-Cell Lung Cancer" was published in 2022. Journal: Comput Math Methods Med.

**Figure 7:** Proportion of VEGF-positive cells in tumor tissues of mice in the four groups. ^∗^Compared with group M, *P* < 0.05; ^#^compared with group C+W, *P* < 0.05.

**Table 1:** Comparison on IHS scores of HIF-1*α* in tumor tissue of mice (*n* = 5, $\overset{¯}{X}\pm S$).

Group	IHS score
Group M	6.00 ± 0.00
Group W	4.00 ± 0.00^∗^
Group C	5.60 ± 0.894
Group C+W	3.20 ± 1.095^∗^^#^

Note: ∗ meant observable difference in contrast to group M; # indicated obvious difference in contrast to group C.

**Table 2:** Comparison on IHS scores of VEGF in tumor tissue of mice (*n* = 5, $\overset{¯}{X}\pm S$).

Group	IHS score
Group M	6.00 ± 0.00
Group W	3.60 ± 0.894^#^
Group C	4.40 ± 0.894^#^
Group C + W	1.60 ± 0.548^∗^

^∗^Compared with group M, *P* < 0.05. ^#^Compared with group C+W, *P* < 0.05.

**Table 3:** Comparison on IHS scores of VEGFR-2 in tumor tissue of mice (*n* = 5, $\overset{¯}{X}\pm S$).

Group	IHS score
Group M	6.00 ± 0.00
Group W	3.60 ± 0.894
Group C	4.80 ± 1.095
Group C+W	2.20 ± 1.095^∗^

^∗^Compared with group M, *P* < 0.05.

## Data Availability

The data used to support the findings of this study are available from the corresponding author upon request.
